# Remote Diagnosis System of Uremia Complicated with Sleep Disorder and Effectiveness of Nursing Intervention

**DOI:** 10.1155/2021/4649139

**Published:** 2021-11-16

**Authors:** Yiqian Wang, Jing Zhu, Jun Cao, Dan Zheng, Lihua Wang

**Affiliations:** Department of Nephrology, The First People's Hospital of Wenling, Zhejiang, Wenling 317500, China

## Abstract

This study aimed to analyze the related factors and remote diagnosis of sleep disorders in patients with uremia and to provide the basis for clinical intervention measures. The Pittsburgh Sleep Quality Index (PSQI) was used to evaluate the sleep quality of 100 patients with uremia. The experimental results show that among 100 patients with uremia, 83 patients (83%) were complicated with sleep disorder, and the average PSQI score was (10.73 ± 1.36). The PSQI score was significantly higher in the elderly, patients with long duration of dialysis, patients with elevated CRP, patients with substandard anemia, and patients with substandard calcium and phosphorus, with statistical significance (*P* < 0.05). The sleep quality of patients with uremia is correlated with depression, age, and penetration age. The worse the sleep quality is, the more severe the depression is. It proved that the sleep quality of dialysis patients is an important factor. *Conclusion*. Sleep disorder is a common complication in patients with uremia. Age, anemia, calcium and phosphorus abnormality, permeation age, and inflammatory status are important factors affecting sleep quality in dialysis patients.

## 1. Introduction

Equipment fault diagnosis technology began in the early 1960s; after nearly 20 years of unremitting efforts, some new technologies (such as information theory, cybernetics, and computer and artificial intelligence) have been continuously introduced into the field of fault diagnosis, and the fault diagnosis technology is constantly enriched and improved [1]. Applications range from simple mechanical equipment diagnosis to diagnosis of aerospace, marine, automotive, water conservancy, and electric power systems, as well as monitoring and control of production processes [2]. Many large systems or critical equipment have been considered in the design stage of the fault diagnosis requirements. The scale of the fault diagnosis system has also developed from the original single machine monitoring system to the present remote distributed monitoring system, so that the monitoring scope of the computer has expanded to the whole enterprise [3]. At present, many enterprises in metallurgy, petrochemical, electric power, and other fields have adopted the equipment remote online monitoring system and achieved remarkable results [4].

Sleep disorder refers to the abnormal amount of sleep and the abnormal quality of sleep, or some clinical symptoms occur during sleep, such as sleep reduction or excessive sleep and sleepwalking [5]. Sleep disorder is a common phenomenon in patients with chronic kidney disease, especially in patients with chronic kidney disease stage 5 maintenance dialysis, with an incidence of 80% [6]. The decline of sleep quality directly leads to the decline of patients' quality of life, with the increasing number of patients with chronic kidney disease caused by diabetes and hypertension, and the increasing number of patients with maintenance hemodialysis, with the improvement of people's demand for quality of life, and sleep disorder has become an urgent problem for patients with chronic kidney disease [7].

Therefore, domestic and foreign studies continue to be conducted. Msosa et al. understood and compared sleep problems and their influencing factors in MHD and PD patients, and it provides theoretical basis for the implementation of corresponding nursing measures, so as to improve patients' sleep quality and dialysis quality of life and improve the long-term survival rate of dialysis patients [8]. Li et al. discussed the clinical effect and nursing key points of hemodialysis patients treated with hemoperfusion and dialyzer in tandem. Eighteen patients were with refractory pruritis, carpal tunnel syndrome, and severe insomnia, and high levels of B2-MG, iPTH, and CRP were treated with HA resin perfusion and dialysis (HP + HD) (treatment group) or hemodialysis (HD) alone (control group) 20 times each. The changes of molecular substances (MMS), serum creatinine, and urea nitrogen were detected before and after treatment. After treatment, small molecules in 2 groups were significantly reduced, and the difference was statistically significant (*P* < 0.05), but the reduction degree of MMS in the treatment group was significantly greater than that in the control group, the difference was statistically significant (*P* < 0.05), and itchy skin, sleep disorder, and appetite were all improved. There was no significant difference in the control group (*P* > 0.05). The HA-type perfusion apparatus and dialyzer in tandem treatment of patients with uremia showed good MMS clearance and improved quality of life [9]. The objective is to investigate the sleep status of uremia patients undergoing maintenance dialysis and analyze its influencing factors, so as to provide theoretical basis for clinical intervention measures. Methods: a total of 187 patients with maintenance dialysis in the department of nephrology of the hospital were selected to study the sleep quality of the patients with the Pittsburgh Sleep Quality Index (PSQI), according to PSQI total score (PSQI ≤ 5 and PSQI > 5), patients were judged to have “good sleep quality” and “poor sleep quality,” and laboratory data and demographic data were collected. Results: (1) 81% of the patients had different degrees of sleep disorder; (2) in elderly patients, patients with long dialysis age, patients with hepatitis, patients with elevated CRP, patients with different beds at night, and patients taking sleeping drugs, the PSQI score was significantly higher, and the difference between groups was statistically significant. (3) PSQI score was significantly correlated with age, BMI, dialysis age, hematocrit, and CRP level; when Hb < 70 g/L, there was a negative linear correlation between Hb and PSQI score. Conclusion: sleep disorders are common in maintenance dialysis patients; age, dialysis age, BMI, and inflammatory status are important factors affecting sleep quality of dialysis patients. When Hb drops to a certain level, sleep quality decreases with the decrease of Hb [10]. On the basis of current research, the analysis of sleep disorder-related factors in patients with uremia and remote diagnosis are proposed to provide the basis for clinical intervention measures. The Pittsburgh Sleep Quality Index (PSQI) was used to evaluate the sleep quality of 100 patients with uremia. The results showed that 83 (83%) of 100 uremia patients were complicated with sleep disorder, and the average PSQI score was (10.73 ± 1.36). The PSQI scores were significantly higher in the elderly, patients with long duration of dialysis, patients with elevated CRP, patients with substandard anemia, and patients with substandard calcium and phosphorus (*P* < 0.05). The sleep quality of patients with uremia is correlated with depression, age, and penetration age. The worse the sleep quality is, the more severe the depression is. Conclusion: sleep disorder is a common complication in patients with uremia. Age, anemia, calcium and phosphorus abnormality, permeation age, and inflammatory status are important factors affecting sleep quality in dialysis patients.

## 2. Data and Methods

### 2.1. Research Object

The subjects of this study were 100 uremic hemodialysis patients admitted to a hospital from October 2019 to November 2020. Exclusion criteria were besides the kidney, it was complicated with other serious medical diseases [11–13].

They were divided into 50 control cases and 50 experimental cases according to the coin toss rule. In the control group, there were 28 males and 22 females with an average age of (55.36 ± 10.69) years, ranging from 40 to 70 years old. Primary disease: 5 cases of hypertensive nephropathy, 7 cases of chronic glomerulonephritis, 5 cases of polycystic kidney disease, 9 cases of diabetic nephropathy. The average time of hemodialysis was (5.27 ± 2.45) years. There were 36 males and 14 females in the experimental group, with an average age of (55.74 ± 10.31) years from 42 to 68 years old. Primary disease: 4 cases of hypertensive nephropathy, 6 cases of chronic glomerulonephritis, 8 cases of polycystic kidney disease, and 12 cases of diabetic nephropathy. The average time of hemodialysis was (6.88 ± 3.72) years. There was no significant difference in equal general data between the two groups, but the comparability was strong (*P* > 0.05) [3].

### 2.2. Remote Diagnosis

Equipment remote diagnosis technology is a combination of equipment diagnosis technology, computer network and communication technology, database, and decision support technology. The University of Michigan is one of the earliest academic institutions to carry out remote diagnosis research abroad; it mainly conducts research on the remote diagnosis and manufacturing system for machining and has set up a propaganda site on the Internet. Westinghouse in the United States can remotely and online monitor the operation of more than 20 power plants in the United States from its diagnostic operation center [14]. Huazhong University of Science and Technology, Xi'an Jiaotong University, Southeast University, University of Science and Technology Beijing, and other units are also carrying out the development and research of the technology. The equipment remote diagnosis system has the following main features:

1. Adopt a variety of network access modes to form a complete enterprise-level diagnosis system to realize real-time monitoring and management of remote equipment; it can grasp and control the state of the equipment in time and accurately, provide reliable technical guarantee for the safe operation of the equipment, and form a nationwide diagnosis network [15].
2. It is conducive to the implementation of diversified collaborative services, realizing real-time consultation of equipment faults between enterprises and remote experts and improving the accuracy and reliability of diagnosis [16].
3. It is conducive to data accumulation and resource sharing, and the remote diagnosis system requires that the data format must be standardized, so as to form a unified database and realize the sharing of diagnosis knowledge and data in a wide range [17].
4. It has good scalability, with the help of Internet/Intranet, the remote diagnosis system can be flexibly extended, and the diagnosis task can be realized on the local area network of several computers in a workshop [18].

### 2.3. Remote Diagnosis Framework

The remote diagnosis system is based on the centralized online monitoring system and distributed online monitoring system, and several central computers are used as diagnosis servers to establish status monitoring points on key equipment [19]. The operation information of mechanical equipment is picked up by the permanently installed sensor at the monitoring point and then input into the field monitoring computer after signal preprocessing and A/D conversion; then, the unit transformation of the signal is carried out to achieve continuous real-time acquisition of device status data and establish remote analysis and diagnosis center in scientific research institutes and universities with strong technical force to provide remote technical support and guarantee for enterprises. By connecting the monitoring points into a complex monitoring network through the network, any monitoring system can make requests for services, upon receiving the request, and the remote diagnostic service center can provide various services and return the diagnosis results. At the same time, the remote service center can also directly obtain the status signals and historical data of the current monitoring points from the Internet, thus forming a complete monitoring system. If a fault occurs on an important device, all the diagnosis resources on the Internet can be mobilized in a short period of time for early diagnosis and timely maintenance, so that enterprises can timely adjust the production process to achieve the purpose of safe and efficient production.

### 2.4. Nursing Methods

All the basic information of the patients, as well as the history and history of allergies to the treatment methods and drugs, should be collected when the control group received routine care and first hemodialysis treatment. In addition, health education and dialysis effect planning, implementation, and evaluation should be carried out before treatment. In addition, weekly diet, exercise, and other nursing plans should be made according to the actual situation of patients. Finally, the self-care knowledge of central venous catheters and internal venous fistulas should be explained to patients.

The experimental group carried out detailed nursing intervention. (1) First, a detailed health record was established for the patients, and the information materials such as the hemodialysis status, digestive function, eating habits, and education level of the patients were recorded. Information should include daily physical activity, blood pressure, urine volume, food intake, and water intake. (2) Second, nursing staff should choose the appropriate way of exercise and diet. Calculate the amount of water, potassium, and protein in food, according to the changes of the patient's daily intake, physical activity, water intake, urine volume, and other indicators, and the patient's diet plan and exercise mode were improved. (3) In addition, complications should be given prevention and treatment of nursing. Caregivers need to teach patients how to deal with common complications. High blood potassium: nursing staff needs to guide patients less or limit the consumption of some vegetables and fruits, such as bananas, laver, and potatoes, and teach patients to learn to use the method of cooking to take out the potassium ion contained in food. Heart failure: the nursing staff should control the patient's blood pressure at 130/80 mmHg and the blood suction rate at 80–10 ml/min before hemodialysis. Internal leakage occlusion: aseptic operation principles should be strictly observed before hemodialysis, and button puncture should be avoided. Rope ladder puncture should be performed according to specific conditions, and buttonhole puncture should be performed in poor conditions. After dialysis treatment, it is necessary to carry out correct compression, guide the patient to check the tremor and vascular fluctuation of the internal fistula every day, and seek medical attention immediately if abnormal conditions are found. (4) Finally, to give psychological support, it is necessary to positively evaluate the psychological changes of patients, timely guide the patients' bad emotions to carry out health education for patients as soon as possible, enhance patients' confidence in treatment, encourage patients to develop interests and hobbies, participate in social activities, divert attention, and keep optimistic and positive attitude.

### 2.5. Nursing Observation Indicators

#### 2.5.1. Methods of Sleep Quality Evaluation

Pittsburgh Sleep Quality Index (PSQI) was used to assess sleep quality. PSQI scale was composed of 7 parts and 19 items. It was a scale for the subjective evaluation of self-sleep quality by patients, with a total score ranging from 0 to 21. The total score >7 indicates poor sleep quality, the higher score indicates poor sleep quality, the score between 0 and 7 indicates good sleep quality. and the score 8–21 indicates poor sleep quality.

#### 2.5.2. Pittsburgh Sleep Quality Index (PSQI)

All subjects were assessed using the Pittsburgh Sleep Quality Index scale (PSQI), and fasting venous blood was collected for clinical biochemical indexes. According to the PSQI scores O–7, they were divided into group A, and 8–21 into group B.

### 2.6. Statistical Methods

All the data were processed by statistical software SPSS18.0, the measurement data (quality of life score) was expressed as (*x* ± *s*), and the *t*-test was performed for comparison: count data (complication rate), rate (%), and the chi-square (*X*^2^) test comparison. The difference was statistically significant (*P* < 0.05).

## 3. The Results

### 3.1. Comparison of Complication Rates between the Two Groups (Table 1)

The incidence of complications in the experimental group was much lower than that in the control group (*P* < 0.05).

### 3.2. Incidence of Sleep Disorders

A total of 110 cases were observed in this study, including 19 cases in group A, 91 cases in group B, and 9L cases with concurrent sleep disorder, accounting for 82.7% of the total cases; the mean PSQI score was (10.73 ± 1.36), indicating that patients with end-stage renal disease were prone to sleep disorders. Univariate analysis showed that the PSQI score was significantly higher in the elderly patients, patients with long dialysis age, patients with elevated CRP, patients with substandard PTH, HB, and patients with substandard calcium and phosphorus (*P* < 0.05), and the difference was statistically significant (*P* < 0.05), as given in Table 2.

### 3.3. Multivariate Logistic Regression Analysis

The results showed that the risk factors for sleep disorders in patients were age ≥60 years, hypercalcium and hyperphosphatemia, substandard PTH, and high CRP. Meanwhile, it was found that the longer the penetration age of patients, the more severe the sleep disorders, as given in Table 3. In addition, the sleep quality of patients was correlated with depression, age, and penetration age. The worse the sleep quality was, the more severe the depression was, as given in Table 4.

## 4. Discussion

As can be seen from Figure 1, hemodialysis not only improves the patient's life expectancy but also improves the patient's quality of life to the maximum extent. The more the complications, the lower the quality of life. Among them, sleep disorder is the common cause of patients with maintenance hemodialysis. Sleep disorder can not only lead to various psychological diseases but also cause the aggravation of physical disease symptoms. But patients with uremia must be treated with maintenance hemodialysis to stay alive, and a study in the United States showed that dialysis patients had more severe sleep disorders; therefore, shortening patients' dialysis may reduce their sleep, that is to say, the longer the dialysis time, the more obvious the sleep disorder; this study also showed that the longer the dialysis age, the more severe the sleep disorder. Nearly 80% of elderly patients on maintenance hemodialysis have severe sleep disorders. There are also a lot of reports abroad that sleep disorder is the common mental state in hemodialysis, and the incidence rate can be as high as 60–80%. The results of this study showed that 83% of the patients had poor sleep quality, and the incidence rate was higher than that reported at home and abroad (60–80%), which was related to the economic level, family, and social burden of the patients in our center. In this study, it was found that the degree of sleep disturbance was significantly correlated with the PSQI score, age, dialysis age, hematocrit, and CRP level.

In the general population, sleep quality declines with age, uremia patients often have abnormal calcium and phosphorus metabolism, and patients with end-stage renal disease often have an inflammatory response. Unruh reported in patients with uremia blood calcium and blood phosphorus levels such as substandard housing that causes itchy skin, bone pain, somatic diseases such as cardiovascular disease symptoms, and further increase in patients with sleep disorders; There are also reports in China that the sleep disorder of uremia patients is significantly related to the prolongation of age, penetration age, and the increase of calcium phosphorus product. Sun Jianjun found in his study that microinflammation in uremia patients is also an important reason for maintaining the sleep quality of hemodialysis patients; our research suggests that the risk factors for sleep disorders in patients were age ≥60 years, hypercalcium and hyperphosphatemia, PTH substandard, and CRP, which were similar to relevant reports at home and abroad. Zhang Jingli and other foreign studies show that sleep quality is positively related to depression and anxiety. Meanwhile, sleep quality affects the mental health and quality of life of patients with uremia to some extent. The results of this study showed that uremia sleep quality was correlated with depression, and the worse the sleep quality was, the more severe the depression was. The sleep quality of hemodialysis patients was positive with depression, and the difference was statistically significant (*P* > 0.05).

## 5. Conclusions

This study aimed to analyze the related factors of sleep disorder in patients with uremia and to provide the basis for clinical intervention. The Pittsburgh Sleep Quality Index (PSQI) was used to evaluate the sleep quality of 100 patients with uremia. The results showed that 83 (83%) of 100 uremia patients were complicated with sleep disorder, and the average PSQI score was (10.73 ± 1.36). The PSQI scores were significantly higher in the elderly, patients with long duration of dialysis, patients with elevated CRP, patients with substandard anemia, and patients with substandard calcium and phosphorus (*P* > 0.05). The sleep quality of patients with uremia is correlated with depression, age, and penetration age. The worse the sleep quality is, the more severe the depression is. Thus, this study concludes that sleep disorder is a common complication in patients with uremia. Age, anemia, calcium and phosphorus abnormality, permeation age, and inflammatory status are important factors affecting sleep quality in dialysis patients.

## Figures and Tables

**Figure 1:** Comparison of sleep quality.

**Table 1:** Comparison of complication rate between the two groups.

Group	High potassium	Hypokalemia	Heart failure	Leak occlusion	Complication rate (%)
The control group (*n* = 50)	6	3	3	2	0.28
The experimental group (*n* = 50)	2	1	1	0	0.08
*X* ^2^					10.4812
*P*					0.0012

**Table 2:** Univariate analysis of general data of patients.

Group	The control group	The experimental group	*P*
Age	49.32 ± 6.74	70.02 ± 9.39	0.001
Through the ages	1.71 ± 0.24	4.43 ± 0.24	0.011
Hemoglobin	102.00 ± 0.31	77.00 ± 0.11	0.011
Blood urea nitrogen	30.12 ± 0.14	30.98 ± 0.18	0.625
Serum creatinine	902.32 ± 132.5	917.78 ± 95.4	0.138
CRP	2.86 ± 0.36	5.87 ± 0.66	0.020
Blood calcium	2.36 ± 0.33	2.71 ± 0.12	0.043
Blood phosphorus	1.36 ± 0.32	2.21 ± 0.23	0.012
PTH	497.0 ± 00.43	834.32 ± 0.32	0.001
Ferritin	198.3 ± 00.25	194.53 ± 0.21	0.220
Kt/V	1.37 ± 0.22	1.39 ± 0.16	0.520

**Table 3:** Multifactor scores of sleep disorders in patients with uremia.

Factors	Evaluation of sleep quality	
	*β*	*P*
Age ≥60 years	2.145	0.001
Through the ages	0.053	0.042
Hemoglobin	2.708	0.001
CRP	0.849	0.001
Blood calcium	2.763	0.010
Blood phosphorus	1.100	0.011
PTH	0.954	0.001

**Table 4:** Linear correlation analysis of age and penetration age with depression and sleep quality in patients with uremia.

Factors	Depression level		Sleep quality score	
	*R* value	*P* value	*R* value	*P* value
Age	0.372	0.20	0.262	0.001
Through the ages	0.289	0.011	0.351	0.010
Depression scores	0.983		0.721	0.001
Sleep quality score	0.721	0.001	0.983	

## Data Availability

The data used to support the findings of this study are available from the corresponding author upon request.
